# Application of CT Medical Imaging Combined with Deep Learning 3D Reconstruction in the Diagnosis and Rehabilitation of Anterior Cruciate Ligament Injury in Table Tennis Players

**DOI:** 10.1155/2021/1152368

**Published:** 2021-12-17

**Authors:** Zhenlei Chen, Jilai Xu, Youqing Shen, Tianshu Zhao, Jiayi Dong

**Affiliations:** ^1^School of Physical Education, Hubei University of Education, Wuhan, Hubei, China; ^2^Graduate School of Medicine, Juntendo University, Tokyo, Japan; ^3^School of Sports Medicine and Physical Therapy, Beijing Sport University, Beijing, China

## Abstract

Because of the intense competition, table tennis requires players to bear a strong physiological load, which increases the risk of sports injury. Anterior cruciate ligament (ACL) is an important structure of the knee joint to maintain forward stability and rotational stability and is also a common sports injury in table tennis players. ACL has poor self-repair ability after injury. Therefore, the purpose of this study is to provide a more comprehensive, reliable, and representative theoretical basis for the diagnosis and rehabilitation of anterior cruciate ligament injury in table tennis players, and three-dimensional reconstruction of ACL using dual-source computed tomography (DSCT) combined with deep learning was conducted. For this purpose, a number of table tennis players with ACL injuries were collected, and each patient underwent arthroscopic anterior cruciate ligament reconstruction. DSCT scanning was performed on several knee joints, the 3D model of the knee joint was reconstructed using a CT image postprocessing workstation, and the medial wall of the femoral lateral condyle was reconstructed, as well as the reconstructed single tract of bony canal, tibial plateau, and bony canal. Then, the Lysholm score was used to score the cases, with scores greater than 75 as the excellent group and below 75 as the poor group. The relative positions of the central points of the femoral and tibial canals were marked and measured. The results were as follows: 3D-CT reconstruction could clearly reflect the situation after anterior cruciate ligament reconstruction. In clinic, it is used to evaluate the relationship between bone tunnel location and graft shape so as to guide the surgeon to improve the operation.

## 1. Introduction

To promote the development of medical technology is the most meaningful help of artificial intelligence to human beings so that machines, algorithms, and big data can serve human health and smart medical treatment will become the core technology for people to resist diseases and prolong their lives in the future. In China, the influence of ACL injury on athletes cannot be ignored, and its incidence has been on the rise. The knee joint anatomical structures and characteristics of it in the human body function position that knee injury to become one of the easiest and most common injuries; however, an ACL injury is the most common in clinic, cruciate ligament plays an important role in maintaining the stability of the knee joint [1–3], and anterior cruciate ligament injury is common. Approximately 200,000 ACL injuries are reported each year in the United States, with approximately 100,000 requiring surgery. According to domestic research reports, the total incidence of anterior cruciate ligament fracture in China is 0.47% (32/6810). Failure to timely and effective repair will cause a series of secondary injuries such as articular cartilage, degenerative changes of the knee joint, and medial and lateral meniscus and seriously affect the function of the knee joint [4]. In addition, due to its own histological characteristics and poor blood supply of the ACL, the central ligament and the bone attachment area of the ligament are deficient in blood supply [5]. Therefore, after the ACL fracture, the original state cannot be restored depending on its own characteristics, which tends to lead to the functional instability of the affected limb [6, 7] and cannot meet the life needs of patients. With the continuous development of arthroscopic surgery, ACL reconstruction is an essential and effective measure in clinical treatment. With the aid of arthroscopy, the method of anterior cruciate ligament reconstruction and location mainly relies on the experience accumulated by surgeons for many years. If the surgeon has a poor experience, hand reconstruction will fail [8, 9]. With the rapid development of 3D-CT and its wide application in various departments in hospitals, clinicians have paid more attention to it because of its features of high scanning speed, time resolution, spatial resolution, rapid imaging, low radiation dose, and stereoscopic visualization for bone tissue. Iriuchishima et al. [10] have used 3D-CT to conduct relevant studies on anatomical footprints of ACL in femur and tibia and achieved certain results. 3D-CT can obtain the volume data of the examined site during a scan, which can carry out three-dimensional reconstruction of various structures in multiple planes, measure the orientation of the center of the femoral and tibial tunnels in three-dimensional space, and analyze the performance of the femoral and tibial tunnels in CT after anterior cruciate ligament rupture reconstruction. According to the Lysholm score, the enrolled patients were divided into the excellent knee function group and the poor knee function group, and there was no significant difference between the femoral and tibial insertion positions of the knee at the operation side between the two groups, so as to explore the imaging parameters reflecting the functional recovery after anterior cruciate ligament reconstruction. Then, the positions of the tibia and femur bone tunnel were measured to study the differences of the positions of the femur and tibia bone canal under different clinical curative effects and the corresponding radiation parameters in order to provide theoretical support for the surgeons in the clinical operation of an anterior cruciate ligament injury in table tennis players in the future.

In this paper, we are going to provide a more comprehensive, reliable, and representative theoretical basis for the diagnosis and rehabilitation of anterior cruciate ligament injury in table tennis players, and three-dimensional reconstruction of ACL using dual-source computed tomography (DSCT) combined with deep learning was conducted. For this purpose, a number of table tennis players with ACL injuries were collected, and each patient underwent arthroscopic anterior cruciate ligament reconstruction. DSCT scanning was performed on several knee joints, and the 3D model of the knee joint was reconstructed using a CT image postprocessing workstation, and the medial wall of the femoral lateral condyle was reconstructed, as well as the reconstructed single tract of bony canal, tibial plateau, and bony canal. Then, the Lysholm score was used to score the cases, with scores greater than 75 as the excellent group and below 75 as the poor group. The relative positions of the central points of the femoral and tibial canals were marked and measured. 3D-CT reconstruction could clearly reflect the situation after anterior cruciate ligament reconstruction. In clinic, it is used to evaluate the relationship between bone tunnel location and graft shape so as to guide the surgeon to improve the operation.

The remaining part of this paper, which is important to highlight, is organized as follows.

In the subsequent section, that is, related work, a brief but comprehensive review of the existing literature is presented where the focus is on sepsis-related diseases. In Section 3, the proposed mechanism is presented, where sophisticated details are provided about various parts of the proposed setup. Experimental results and observations were presented in Section 4. A general discussion about the proposed method and its applicability is provided. Finally, concluding remarks and future directives are provided in the last section.

## 2. Related Work

Artificial intelligence has been gradually developed since the mid-1960s by the pursuit of universal, general research into specific studies, general problem-solving strategies, and specific areas of professional knowledge and practical experience, produced by the expert system based on knowledge of all kinds of artificial intelligence systems and the artificial intelligence to the society towards practical application research. In 1965, E.A. Eigenbaum opened up a new field of artificial intelligence research called expert systems, reclaiming the concept of “knowledge is power.”

Wang Jun believes that sports risks always exist and can be avoided. The way, content, intensity, sports level, health level of athletes, and the depth of their knowledge of sports are all related to the probability of sports risks [11]. Table tennis is a kind of antinet sport; the players swing the ball with speed, rotation, strength, arc, and landing point. With the continuous development of the overall level of table tennis in the world and the constant change of competition rules, table tennis has changed in terms of material and size. When the diameter of the table tennis ball changed from 38 mm to 40 mm, the speed of the ball decreased by 23% and the rotation of the ball decreased by 13%. Therefore, when the diameter of the ball becomes larger, the speed and rotation of the ball will be reduced. Athletes need better ball holding ability and physical quality to adapt to these changes. The nonblocking serve also requires athletes to have higher holding ability and better physical fitness. Chu also mentioned the use of inorganic glue; table tennis players need to have a better ability to hold; at the same time, the inorganic glue makes the racket flexibility greatly reduced; then, the athletes must increase the range of hitting action. The implementation of the 11-point game system requires athletes to be more energetic and active when playing every point, so they also need higher physical fitness [12, 13].

ACL injury is one of the common knee injuries at present, accounting for about 40% of sports injuries [14]. Scholars led by Kazunori Yasuda and Freddie Fu proposed the concept of ACL anatomical reconstruction. ACL under arthroscopy revascularization has become the main treatment of knee ACL rupture, the bone position is one of the key factors for the successful operation of anterior cruciate ligament reconstruction [15], and the error of the femur and tibia bone position will cause abnormality of the biomechanics of the knee joint, which affect the rotation of the knee joint stability and before and after stretching movement lead to joint degeneration or secondary damage to cartilage and meniscus. However, it is very difficult to establish the “correct” bony canal. Studies have shown that the error rate of femoral canal localization reaches 25%∼65% [16] because it is difficult to accurately distinguish the stump of the ligament in knee joints with chronic ACL injuries. In an anatomical study of anterior cruciate ligament, Siebold et al. [17] measured the femoral insertion area of ACL in femur specimens: male 98 ± 22 mm^2^ and female 76 ± 13 mm^2^; long axis: male 15.2 ± 2 mm and female 14.3 ± 3 mm; short axis: male 8.4 ± 2 mm and female 7.8 ± 2 mm. Yasud et al. [18] found in their study that the center of the femur insertion of the posterior external band was 5–8 mm away from the inferior cartilage margin of the femur at the position of 90 degrees of knee bend. Mochizuki et al. found that the femur insertion of the anterior internal band and a posterior external band of the ACL of the left knee were located at 1 : 40 and 3 : 10. ACL tibial insertion is located in the tibial plateau, and its anatomical signs are mainly divided into bone and soft tissue signs. As for the anatomical markers of tibial insertion, previous studies are not completely identical. The results showed that the length and width of tibial insertion were 14 ± 2 mm and 9 ± 1 mm, respectively. Some studies measured the tibial insertion size by arthroscopy, and the results showed that the AMB length was 9.2 ± 1.2 mm, and the width was 8.9 ± 0.9 mm. PLB length is 7.1 ± 1.1 mm, width is 6.9 ± 1.0 mm, and the total length of ACL tibial insertion was 16.5 ± 2.0 mm. In studies on anterior cruciate ligament positioning methods, quadrant method (four-grid method), AMIS method, intercondylar fossa clockwise positioning method, and Takahashi method were mainly used for femoral lateral positioning. Woo et al. [19] conducted a cadaver study and reconstructed the ACL at the standard 11 o'clock of the right knee (1 o'clock of the left knee member). The forward stability of the hepatic bone was recovered satisfactorily, but the control effect of rotation stability was poor. Zhao Bin et al. positioned the femoral tunnel at 1∼2 points of the left knee and 10∼11 points of the right knee and achieved good results in postoperative follow-up. In recent years, it has been reported that ACL reconstruction using Western blotting anatomical center point can better restore the forward and rotational stability of the knee joint, which can be used as a theoretical basis for reconstruction. Ferrtti et al. [20] found in the study of 8 knee joints that the anterior angle of the lateral meniscus of 3 knee joints was located in front of the tibial insertion, among which 2 were located in front of the midpoint of AMB and ACL, and 1 was located in the same sagittal position as the midpoint of AMB. There are many studies on PCL as a localization marker for tibial insertion during ACL reconstruction, and it is also a very important localization marker because it is easy to find intraoperatively. Hutchinson and Bae studied the anatomy of 42 pairs of knee joints and obtained the distance between the ACL posterior edge and PCL (6.7 ± 1.2 mm) and the distance between the ACL midpoint and PCL (10.4 ± 2.4 mm) with the guide assisted X-ray measurement. Heming et al. observed 12 frozen knees with different knee bend angles, measured that the midpoint of ACL was 15.0 mm in front of PCL, and concluded that the knee bend angle not only had no significant influence on the distance before ACL and PCL but only had a certain influence on the length of the tibial canal. Purnell et al. [21] studied 8 knee joints through 3D reconstruction and arthroscopic exploration and measured the distance between the posterior edge of ACL and the leading edge of PCL (16.5 ± 2.1 mm).

Siemens SOMATOM definition system is a dual-energy computed tomography 3D imaging (DSCT) system developed by Siemens in Germany for the medical field. It is well known that conventional CT has advantages in showing bony structures but has significant disadvantages in soft tissue imaging. Traditional CT machines only install one X-ray transmitter and one receiver. DSCT adds a set of ray transmitting and receiving devices on the basis of traditional CT. Equipped with two sets of X-ray sources A and B, DSCT can emit rays of two different energies for scanning, namely, dual-energy scanning. The system separates and integrates two sets of scan data at different energies to identify structures that cannot be identified by conventional CT. The development of DSCT has expanded the scope of new clinical applications. This technique can be applied to the 3D reconstruction of the coronary system, gastrointestinal system, blood vessels, bone tendon, and so on. Yasumoto et al. have used DSCT to study the regeneration of donor semitendinosus muscle after ACL reconstruction, which can clearly display the residual shape of postoperative semitendinosus muscle. This study is our first attempt to use DSCT to reconstruct ACL graft images and successfully display the morphological structure of postoperative ACL grafts in a three-dimensional manner. LohanDG et al. believed that when scanning tendons and ligaments with DSCT, patients received a significantly higher dose of gamma ion radiation than single-source CT. Although the scanning rate of DSCT is increased, the double bulb requires two exposures, increasing the dose of X-rays received by the subject.

## 3. Proposed Method

### 3.1. 3D Reconstruction Technology Based on Deep Learning

#### 3.1.1. Convolutional Neural Network

Object 3D reconstruction can be realized by using a neural network, so it is necessary to learn the basic theory of the neural network. In recent years, many computer problems have made good progress through convolutional neural networks. Convolutional neural network consists of a convolutional layer, pooling layer, and full connection layer. The convolutional layer is the most important part of the convolutional neural network. Each neuron node is only connected to a part of the upper layer of neurons, and the size of the connected area is the size of the filter, commonly known as the receptive field. The size of the filter is artificially set. Commonly used filter sizes are 3 × 3 or 5 × 5, and the depth of the filter is the same as the depth of the input data. During the convolution operation, in addition to the filter size *f* × *f*, the number of filters *k*, the convolution step size *s*, and the padding size *p* need to be specified. Assuming the input image of *n* × *n* size, the output matrix size of the convolution layer is

(1) $$\begin{array}{c} \left[\frac{n+2p-f}{s}+1\right]\times \left[\frac{n+2p-f}{s}+1\right]\times k. \end{array}$$

In the neural network, the linear weights of nodes and weights of the upper layer are the outputs of the upper layer and then passed to the neurons of the next layer through an activation function. If the activation function is not used, then the nodes of each layer have a linear relationship with the nodes of the upper layer. No matter how deep the layers of the neural network are, the output of the neural network is a linear combination of inputs, which is the same as the effect without hidden layers, and the expression ability of such a network is limited. Therefore, the activation function is usually nonlinear, and the neural network of the activation function is introduced. As the number of neural network layers increases, the learning ability is enhanced. The earliest neural networks usually use the sigmoid function or Tanh function as the activation function. In recent years, neural networks have widely used the ReLU function and the improved ReLU function.

The sigmoid function was the most commonly used activation function in the early days, with the following formula:

(2) $$\begin{array}{c} f\left(z\right)=\frac{1}{1+e^{-z}}. \end{array}$$

The formula for the Tanh function is as follows:

(3) $$\begin{array}{c} \tanh\left(x\right)=\frac{e^{x}-e^{-x}}{e^{x}+e^{-x}}. \end{array}$$

The Tanh function solves the problem that the sigmoid function is not zero-centered output. However, the derivative of the Tanh function is still in the saturated region, and the problem of gradient disappearance cannot be solved. And, you still have powers of the Tanh function. The ReLU activation function is defined as follows:

(4) $$\begin{array}{c} f\left(x\right)=\max\left(0,x\right). \end{array}$$

From the above equation, it is not difficult to see that the ReLU function is a piecewise linear function. If the input is negative, the output is 0, while if the input is positive, the output is equal to the input. Therefore, the ReLU function achieves unilateral suppression. Unilateral inhibition of ReLU function results in sparse activation of neurons in the neural network, and some neurons in the network may never be activated. The advantage of the ReLU function is that there is no power function, the calculation speed is fast, and the convergence speed is faster.

Leaky ReLU has emerged to solve the “Dead ReLU” problem of the Leaky ReLU function, which is defined as follows:

(5) $$\begin{array}{c} f\left(y\right)=\max\left(\varepsilon y,y\right), \end{array}$$

where *ε* is the slope factor, usually a small gradient value. Unlike ReLU, the Leaky ReLU function does not set negative values to zero in order not to lose all negative information.

#### 3.1.2. Three-Dimensional Convolutional Neural Network

The 3D convolutional neural network is often used to extract features of 3D image data or classify features of 3D image data and is often used in the medical field and video processing field. This section introduces the 3D convolution layer and 3D pooling layer. It is assumed that the size of the input data is *a*_1_ × *a*_2_ × *a*_3_, the number of channels is *c*, the size of the convolution kernel is *f*, that is, the dimension of the convolution kernel is *f* × *f* × *f* × *c*, the number of filters is *k*, the size of the convolution step is *s*, and the padding is *p*. The final output of three-dimensional convolution is

(6) $$\begin{array}{c} \left[\frac{a_{1}+2p-f}{s}+1\right]\times \left[\frac{a_{2}+2p-f}{s}+1\right]\times \left[\frac{a_{3}+2p-f}{s}+1\right]\times f. \end{array}$$

When the 3D pooling layer adopts the maximum value for sampling, it is assumed that the size of the input data is *a*_1_ × *a*_2_ × *a*_3_, the number of channels is *c*, the size of the convolution kernel is *f*, that is, the dimension of the convolution kernel is *f* × *f* × *f* × *c*, and the convolution step is *s*. The output of the maximum 3D pooling layer is

(7) $$\begin{array}{c} \left[\frac{a_{1}-f}{s}+1\right]\times \left[\frac{a_{2}-f}{s}+1\right]\times \left[\frac{a_{3}-f}{s}+1\right]. \end{array}$$

#### 3.1.3. 3D Reconstruction Technology Based on Deep Learning

The 3D reconstruction network based on deep learning can learn from a large amount of data to map 2D images of objects to 3D geometric structures. The process of realizing 3D reconstruction technology based on deep learning is shown in Figure 1. By entering the two-dimensional images and training deep neural network, 3D data is output. After it, the output of 3D data loss function is calculated with real 3D data, backpropagation algorithm, and gradient value. Meanwhile, gradient descent method is used to update the parameters in the model, after several iterations, to predict three-dimensional data model.

#### 3.1.4. Loss Function

In deep learning, models are solved and evaluated by minimizing loss functions. This section mainly studies the cross-entropy loss function, Lovasz-Softmax, and other loss functions. The cross-entropy loss function is usually used for classification problems. In the binary classification problem, the prediction results of the model are only 0 and 1. Assuming that the probability of prediction is *p*, then the probability of prediction is 1-*p*. The calculation formula is as follows:

(8) $$\begin{array}{c} L=\frac{1}{N}\underset{i}{\sum }L_{i}=\frac{1}{N}\underset{i}{\sum }-\left[y_{i}\log\left(p_{i}\right)+\left(1-y_{i}\right)\log\left(1-p_{i}\right)\right], \end{array}$$

where *y*_*i*_ refers to the label of sample *i*, *y*_*i*_ of positive sample is 1, *y*_*i*_ of negative sample is 0, and *p*_*i*_ is the probability that the sample is positive.

To apply the cross-entropy loss function to the network training designed in this section, it should be defined as the sum of voxel cross entropy. Each individual element (*i*, *j*, *k*) of final output in line with the Bernoulli distribution [1 − *p*(*i*, *j*, *k*), *p*(*i*, *j*, *k*)], the corresponding real output *y*(*i*, *j*, *k*)*ε*{0,1}, and the sum of the voxel cross-entropy formula is as follows:

(9) $$\begin{array}{c} L\left(x,y\right)=\underset{i,j,k}{\sum }-\left[y_{\left(i,j,k\right)}\log\left(p_{\left(i,j,k\right)}\right)+\left(1-y_{\left(i,j,k\right)}\right)\log\left(1-p_{\left(i,j,k\right)}\right)\right]. \end{array}$$

Lovasz-Softmax loss function is a kind of IoU-based loss function. In the image segmentation problem, the Lovasz-Softmax loss function is better than the cross-entropy loss function. IoU is used as an evaluation index in this paper, so the Lovasz-Softmax loss function is used in the network studied in this paper. Lovasz-Softmax is calculated as follows:

(10) $$\begin{array}{c} m_{i}\left(c\right)=\left\{\begin{array}{cc} 1-f_{i}\left(c\right) & \text{if }c=y_{i}^{*}\\ f_{i}\left(c\right) & \text{otherwise} \end{array}\right),\\ \text{loss}\left(f\left(c\right)\right)=\bar{\Delta_{J_{c}}}\left(m\left(c\right)\right). \end{array}$$

### 3.2. Probabilistic Neural Network (PNN)

PNN network is a kind of feedforward neural network, which is evolved from a radial basis function network, and its theoretical basis is the Bayesian minimum risk criterion. PNN networks constitute the nearest classifier when the SPREAD value of distribution density is close to 0. When the SPREAD value is large, it constitutes a neighbor classifier for several training samples. The hierarchical model of PNN is composed of four layers: input layer, pattern layer, summation layer, and output layer. In some pieces of literature, the pattern layer is called the hidden layer, and the summation layer is called the competitive layer. The input layer is responsible for introducing *n* sample feature vectors into the network, and the number of neurons is equal to the dimension of the sample vector. Connection weights connect the pattern layer to the input layer. In order to get the output value of the pattern layer, the similarity between the input feature vector and each mode in the training set should be calculated, and its distance should be calculated by the Gaussian function. The number of neurons in the pattern layer is equal to the number of input sample vectors; that is, there are as many neurons as there are samples. The output of each pattern unit in the pattern layer is

(11) $$\begin{array}{c} f\left(X,W_{i}\right)=\exp\left[\frac{{\left(X-W_{i}\right)}^{T}\left(X-W_{i}\right)}{2\delta^{2}}\right], \end{array}$$

where *W*_*i*_ is the weight of the connection from the input layer to the mode layer; *δ* is the smoothing factor, which plays a crucial role in classification.

### 3.3. Data Collection

#### 3.3.1. Study the Image

A questionnaire survey was conducted, and a number of national table tennis players with ACL injuries of grade II and above were selected. All the patients were diagnosed by past medical history, present medical history, physical examination, and auxiliary examination. Inclusion criteria were as follows: patients aged 15–30 years, surgical indications are clear, and the patient was repaired with a single knee ligament graft. The patient has been informed of the entire treatment process and signed relevant informed documents. Exclusion criteria were as follows: patients with no clear injury history before surgery; imaging examination that does not support the disease; patients with other diseases of the knee joint.

#### 3.3.2. Proposed Research Methods

  Knee function assessment: Comparison was performed according to certain grading standards before anterior cruciate ligament reconstruction; commonly used standards are Tegner motion rating and Lysholm rating. Modeling and measurement methods: all patients underwent CT scan (SOMATOM definition Flash) within 7 days after reconstruction. All patients were examined in a supine position. Postoperative tibial CT examination of all patients can obtain images of various parts of the knee. The examined images are processed professionally, often using multiplane reconstruction (MPR), curved surface reconstruction, three-dimensional volumetric imaging, and surface reconstruction. The multiplanar multidirectional reconstruction shows the anterior cruciate ligament (ACL) in the femoral and tibial bone tunnels and the intra-articular alignment of the ACL. Lateral femoral canal parameters were measured on the reconstructed image of the femur using the quadrant method. On the reconstructed image, the apex line of the intercondylar fossa could be clearly displayed. The total length of the intersection point AB between the apex line of the intercondylar fossa and the anterior and posterior boundaries of the lateral femoral condyle was taken as the apex line length of the intercondylar fossa *e* is the percentage of AB from a distance between the anterior cruciate ligament at the midpoint O of the femoral tunnel and the intersection A of the apex line of the intercondylar fossa and the anterior lateral condyle of the femur. CD is the maximum diameter of the anterior and posterior margins of the tibial plateau, and *f* is the length from the center P of the tibial bone tunnel to the anterior boundary of the tibial plateau. All imaging data were measured twice, and the final results were averaged.
  Follow-up after reconstruction: A small number of table tennis players in this study were lost to follow-up due to some reasons, accounting for about 12% of the total number of cases. The remaining patients received regular follow-up of 6 to 10 months, accounting for approximately 88% of the cases, and all patients were followed for an average of 8 months from study start to study end. Patients were followed up in various forms, mainly by telephone return visit and outpatient examination combined. Questions were asked about the degree and intensity of exercise the patient could achieve, and the knee function was assessed according to the Lysholm score and Tegner exercise rating. The abovementioned patients can be divided into excellent group and poor group by Lysholm score. Lysholm score in excellent group is >75 and Lysholm score in poor group is <75.

### 3.4. Statistical Analysis

All data in this study are from the ADNI1 data set, and the statistical software SPSS21.0 is used for data processing. For statistical data, measurement data were expressed as *x* ± *s*, and counting data were expressed as percentage. Independent sample *t*-test and paired sample *t*-test were used for intergroup and intragroup comparisons, respectively. Count data were tested by *x*^2^ test. *P* < 0.05 was considered as a significant difference.

## 4. Experiments and Results

### 4.1. Model Establishment Based on PNN Neural Network

PNN network design process is shown in Figure 2. A probabilistic neural network as a kind of RBF network, suitable for pattern classification, not only is simple in structure, training, and concise but also can use a linear algorithm to solve the nonlinear problem and has high precision; it is a network to form the strong fault tolerance ability and adaptive ability of diagnosis network system structure and improve the diagnostic accuracy. The research field of this paper is the classification and diagnosis of diabetes, which requires high diagnostic accuracy and fast diagnosis rate. Therefore, PNN neural network is selected to conduct modeling and analyze simulation results.

Firstly, input data was established as the feature vector that could describe ACL. Secondly, the PNN network was created. Training levels and test sets were randomly generated based on the collected medical record data of ACL injury in proportion, of which 75% were used for training and 25% for testing. By analyzing the diagnostic effect of PNN, it can be concluded that the PNN model can successfully classify data samples. After 15 times of training of the PNN network model, the average accuracy reaches 95.6%, so it is feasible to apply PNN to the classification and diagnosis of diabetes (see Table 1 and Figure 3).

### 4.2. Results of the Questionnaire Survey on Athletes' Basic Information

Through the collation and analysis of the survey data, the corresponding research results are obtained. Basic information of table tennis players with an ACL injury is shown in Table 2.

As can be seen from Figure 4, among all the athletes surveyed, ACL injuries occurred during the special training period, accounting for 41.4% of the total number of injuries; occurred in competition period, accounting for 29.8% of the total number of injuries; occurred in the physical training period, accounting for 13.1% of the total number of injuries; occurred in individual training period, accounting for 9.5% of the total number of injuries; occurred in other periods, accounting for 6.2% of the total number of injuries.

The main causes of ACL injury in table tennis are as follows: muscle power imbalance is the first factor; lack of flexibility accounted for the second place; unreasonable use of technology factors accounted for the third place; inadequate preparation activities accounted for the fourth place; lack of self-protection and excessive fatigue in table tennis injury causes ranked the fifth place, as shown in Figure 5.

### 4.3. Comparison of Clinical Data between the Two Groups

There was no significant difference in gender, age, injury type, Lysholm score before reconstruction, and Tegner grade before reconstruction between the excellent group and the poor group ( *P* > 0.05), indicating comparability (see Table 3 and Figure 6 and 7).

### 4.4. Functional Scores of Patients before and after Reconstruction

Among the athletes included in the study, the lowest and highest Lysholm scores were 30 and 80, respectively, and the mean score of all patients was 45.98 ± 14.27. The Tegner grade was 1 at the lowest level and 5 at the highest level, with an average grade of 2.55 ± 0.93. None of the patients had failed surgery or received a second operation. After reconstruction, the Lysholm score ranged from 58 to 100, with an average of 88.03 ± 7.87 points. The lowest Tegner grade was grade 3, and the highest Tegner grade was grade 8, with an average grade of 5.41 ± 2.04. The Lysholm score and Tegner grading of the affected knee joint were significantly better before and after the operation ( *P* < 0.01) (Table 4). In the CT reconstruction data of all patients, the percentage of the projection point on the Blumensaat line of the femoral canal from the anterior condyle of the lateral femur was 45.26%–86.35%. At the other end of the ligament, the length from the center of the tibial canal to the anterior border of the tibial plateau accounted for 27.68%–49.30% of the maximum diameter of the anterior and posterior margins of the tibial plateau, with an average of 68.73 ± 6.86% and 40.27 ± 3.10%, respectively.

### 4.5. Comparison of Insertion Positions of Femur and Tibia

The comparison of bone canal center points (E, F) at both ends of the postoperative ligament of the affected side of the knee between the two groups showed a significant difference (*P* < 0.05), as shown in Figure 8.

## 5. Conclusion

The effect of the operation includes many factors, among which the precise location of the starting and ending point of the ligament is the key to the postoperative effect. Anatomical reconstruction of ACL is to restore its natural form as much as possible. There are various factors leading to the wrong positioning of the bone canal at both ends of the ligament, mainly related to the field of vision of arthroscopic equipment and individual differences and so on. Due to the above reasons, the theoretical positioning knowledge cannot be well applied in clinical practice, so it is difficult to accurately locate the position of the bone canal with only theoretical anatomical knowledge. With the wide application of 3D-CT in clinical practice, its advantages have gradually emerged. After the CT scan, the data will be transmitted to the workstation. With certain technical means, we can arbitrarily remove the tissues we think are not needed, so that the parts we need can be clearly displayed, and through the preoperative evaluation of all parameters, we can do in the process of surgery to know, with ease. In this study, the position of the anterior cruciate ligament in the femoral and tibial bone canal was reconstructed by 3D-CT reconstruction technology, and the conclusions were drawn through statistical analysis. The knee function of patients with anterior cruciate ligament rupture after reconstructive surgery was significantly improved compared with that before surgery. The location of the femoral tunnel has a significant effect on the postoperative efficacy after reconstruction, while the location of the tibial tunnel has no significant effect on the postoperative efficacy. 3D-CT three-position reconstruction technology of knee joints can clearly and intuitively display the bone tissue, which is beneficial for the operator to make the surgical plan. 3D-CT knee reconstruction technology can provide a more comprehensive, reliable, and representative theoretical basis for the diagnosis and rehabilitation of ACL injury in table tennis players.

## Figures and Tables

**Figure 1:** The flow of 3D reconstruction technology.

**Figure 2:** PNN network design process.

**Figure 3:** Accuracy of 15 experiments.

**Figure 4:** The occurrence period of ACL injury.

**Figure 5:** Main causes of ACL injury.

**Figure 6:** Lysholm score before ACL reconstruction in the two groups.

**Figure 7:** Tiger classification before ACL reconstruction of two groups.

**Figure 8:** Comparison of insertion positions of femur and tibia (*x* ± *s*, %).

**Table 1:** PNN network model accuracy.

Methods	Average accuracy	Standard deviation of accuracy
PNN network model	95.6	1.15

**Table 2:** Basic information table.

Age	The training of	Height	Weight	Gender
19 ± 5	10 ± 4	172 ± 15	60 ± 10	Male
19 ± 5	10 ± 4	160 ± 7	55 ± 6	Female

**Table 3:** General information of patients with ACL reconstruction in the two groups.

Group	Good group	Poor group
Gender (male/female, %)	40%/25%	20%/15%
Age (years)	16–25(38.4)	18–28(32.1)
Type of injury (acute/chronic, %)	30%/35%	18%/17%

**Table 4:** Knee joint before and after reconstruction (*x* ± *s*, min).

Project	Before reconstruction	After the reconstruction
Lysholm scale	45.98 ± 14.27	88.03 ± 7.87
Tegner classification	2.55 ± 0.93	5.41 ± 2.04

## Data Availability

The datasets used during the current study are available from the corresponding author on reasonable request.
